# Comparison of Effect of Three Different Surgical Procedures on Ankle Joint Function Rehabilitation of Patients with Hepple V Talus Osteochondral Injury

**DOI:** 10.1155/2022/8110557

**Published:** 2022-10-10

**Authors:** Zhanhua Ma, Junde Wu, Jinglu Han, Yanzhao Hu, Qian Li

**Affiliations:** ^1^Hand and Foot Surgery, Beijing University of Chinese Medicine Third Affiliated Hospital, China; ^2^Sports Medicine, Cangzhou Hospital of Integrated TCM-WM Hebei, China; ^3^General Medicine, Beijing University of Chinese Medicine Third Affiliated Hospital, China

## Abstract

**Objective:**

To discuss and compare the effects of three different surgical procedures on ankle function rehabilitation of patients with Hepple V talus osteochondral injury.

**Methods:**

A total of 60 patients with Hepple V talus osteochondral injury admitted to our hospital from January 2020 to January 2021, among which 17 patients in study group 1 received microfracture surgery, 20 patients in study group 2 received osteochondral autologous transplantation, and 23 patients in study group 3 received with periosteal iliac bone transplantation. The range of motion (ROM) of the patients' angle was evaluated by the goniometer before and after the treatment. The ankle function was evaluated by the ankle-hindfoot score of American Orthopedic Foot and Ankle Society (AOFAS). The ankle joint pain was evaluated by visual analogue score (VAS). The surgical efficacy was evaluated 12 months after surgery, and complications and nursing satisfaction were observed and recorded.

**Results:**

There was no significant difference in ROM, AOFAS score, and VAS score among the three groups before the treatment (*P* > 0.05). ROM and AOFAS score of the three groups were improved, and VAS score was decreased at 6 months and 12 months after treatment (*P* < 0.05). ROM and AOFAS score of group 2 and group 3 were higher than those of group 1, while the VAS score was lower than that of group 1, indicating significant difference (*P* < 0.05). There was no significant difference in ROM, AOFAS, and VAS score between group 2 and group 3 (*P* > 0.05). The surgical efficacy of group 2 and group 3 was higher than that of group 1, indicating statistical significance (*P* < 0.05), while there was no significant difference in the surgical significance between group 2 and group 3 (*P* > 0.05). There was no significant difference in complication rate among the three groups (*P* > 0.05), and the treatment satisfaction of group 2 and group 3 was higher than that of group 1, indicating statistical significance (*P* < 0.05), but there was no significant difference between group 2 and group 3 (*P* > 0.05).

**Conclusion:**

Three different surgical procedures have good therapeutic effect for Hepple V talus osteochondral injury. Osteochondral autologous transplantation and periosteal iliac bone transplantation can reduce the pain of ankle joint, promote the effect of ankle joint function recovery, which can effectively improve patient satisfaction. It is suggested to choose the surgical procedure according to the actual situation of patients.

## 1. Introduction

As a common foot and ankle injury, talus osteochondral injury involves articular cartilage and subchondral bone, and the ankle joint is often accompanied with swelling, pain, flexion and extension disorders, and other symptoms, mainly diagnosed as Hepple V [1]. Even though elaborate knowledge exists concerning ODs of the talus, its etiology and pathogenesis are still not fully understood. Increasing attention is paid to invasive and sometimes expensive surgical treatments, while research for pathogenesis of the lesions has somewhat been neglected. In order to treat ODs in all its dimensions, more should be known about their natural history. The development of an OD may have a sudden onset, but the development of a subchondral cyst is most often a slow process.

At present, surgical treatment is mainly adopted for the treatment of Hepple V talus osteochondral injury, including microfracture surgery, osteochondral autologous transplantation, and periosteal iliac bone transplantation as the main surgical procedures [2, 3]. The above three procedures have been widely used in clinical practice [4, 5]. Therefore, microfracture surgery, osteochondral autologous transplantation, and periosteal iliac bone transplantation were performed, respectively, for the patients with Hepple V talus osteochondral injury in this study, to explore the effect of different surgical procedures on ankle function rehabilitation and surgical efficacy.

## 2. Data and Methods

### 2.1. General Data

A total of 60 patients with Hepple V talus osteochondral injury admitted to our hospital from January 2020 to January 2021 were selected, among which 17 patients in study group 1 received microfracture surgery, 20 patients in study group 2 received osteochondral autologous transplantation, and 23 patients in study group 3 received with periosteal iliac bone transplantation. The patient data are shown in Table 1, indicating no statistical significance (*P* > 0.05) in difference comparison. This study has been reviewed and approved by the Ethics Committee of the hospital.

### 2.2. Inclusion and Exclusion Criteria

#### 2.2.1. Inclusion Criteria

(1) Chronic ankle pain has affected daily life and work of patients. (2) MRI result confirmed that Hepple V talus osteochondral injury was caused by subchondral cyst, and the patient was admitted to hospital for surgical treatment. (3) The diameter of osteochondral defect area ranged from 10 mm to 20 mm. (4) After being informed of the research content by medical staff, the patients and their relatives participated voluntarily.

#### 2.2.2. Exclusion Criteria

(1) Hepple stage I–IV talus osteochondral injury. (2) Severe osteoarthritis, ankle deformity, poor force line of affected limb, severe osteoporosis, and other diseases. (3) Mental disorder and retardation, inability to communicate normally.

### 2.3. Surgical Procedure

#### 2.3.1. All Patients Received General Anesthesia as Reported Previously [5]

Group 1 received microfracture surgery. The patient was assisted to lie at supine position cushioned with the iliac pillow. The tourniquet was tied at the proximal end of the femur on the affected side, maintaining the pressure at 30 mmHg for 60 min. With lateral and anteromedial surgical approaches, the internal and lateral sulcus and tibiotalar joint were examined successively. It cleaned up the proliferative synovial tissue and osteophyte and found out the cartilage lesion, cleaned out the unstable cartilage that was fallen off and softened, and removed the necrotic tissue and sclerotic wall in the subchondral bone cyst with a scraper. Then, drilled vertically with the microfracture processor at a depth of 5 mm and a spacing of 3 mm. After drilling, the tourniquet will be loosened to observe the bleeding of the drilling hole. If the blood oozed evenly, the drilling is appropriate.

Group 2 received osteochondral autologous transplantation. The hyperplastic synovial tissue and osteophyte were examined and cleaned out by arthroscopy. After debridement or lifting the cartilage, the medial malleolus was osteotomized and turned downward to expose the talus lesion. With the help of osteochondral autologous transplantation system, a vertical drilling hole was made at a depth of 10 mm. The T-shaped handle should be selected at a uniform speed to remove the osteochondral column in the lesion area completely. A longitudinal incision of 5 cm was made beside the medial patella to expose the nonweight bearing area of the medial patellofemoral articular surface of the femoral condyle. Then, the osteochondral column with hyaline cartilage was taken out by a drill with the same size as the talus lesion area. The osteochondral cartilage was carefully inserted into the bone groove of the lesion area and pressed tightly. The two cartilage surfaces should be at the same level. After the impact was eliminated by flexion and extension of ankle joint, two cannulated screws were inserted to fix the medial malleolus.

Group 3 received periosteal iliac bone transplantation. The hyperplastic synovial tissue and osteophyte were cleaned out by arthroscopy. After debridement or lifting the cartilage, L-shaped osteotomy was performed on the medial malleolus to expose the inner and upper part of the talus. The cystic lesion was located by Kirschner wire, and the columnar bone groove was made perpendicular to the cartilage surface with the trephine to remove the subchondral cystic lesions. Kirschner wire was used to drill holes at the bottom and side of the cystic sclerosis. A trephine with the same diameter as the talar lesion area was selected to remove the iliac bone lock, with the length of the iliac bone lock slightly shorter than that of the lesion bone column, and the surface periosteum should be preserved. At the same time, a proper amount of cancellous bone was removed from the iliac crest and placed at the bottom of the bone groove of the talus, which was pressed firm and then inserted into the bone lock. The periosteum on the surface of the iliac bone should be basically level with the surrounding articular cartilage, and the medial malleolus was fixed with two cannulated screws.

The patient can be assisted with passive ankle flexion and extension 7 days after operation, for 3 times a day and 10 minutes each time. The patient can have rehabilitation training with the help of passive continuous activity and passive assisted exercise and receive ice compress after each exercise. No weight bearing is allowed within 42 days after operation. Partial weight bearing exercise can be carried out from 49 to 56 days after operation. Ankle X-ray examination should be performed 63 days after operation. Full weight bearing is possible if the fracture line is blurred. Strenuous activity is strictly prohibited within 90 days after operation.

### 2.4. Observation Indexes

The range of motion of ankle joint was measured and compared before and after treatment with goniometer. The stress, contact state, and displacement of each component of the ankle joint were observed in the different groups to determine its maximum value and location. The maximum pressure was recorded as the experimental data and analyzed to obtain the column diagram, and the changes in pressure were discussed. In this study, the primary outcome was a displacement of the talus and contact pressure of the articular surface. Secondary outcomes were equivalent stresses of the proximal talus, tibial cartilage, and talus cartilage.

50 points or below of AOFAS score represent poor, 51-74 points represent average, 75-89 points represent good, and 90-100 points represent excellent.

The ankle pain was evaluated by VAS score before and after treatment. VAS score ranged from 0 to10, 0 for no pain, 1-3 for mild pain, 4-6 for moderate pain, 7-9 for severe pain, and 10 for severe pain that is unbearable.

The surgical efficacy was evaluated and compared one year after operation. After treatment, the pain symptoms of patient were significantly relieved, ankle joint function was significantly improved, and MRI results showed that edema disappeared or cystic changes, which represented an effective case. After treatment, patient had no improvement in clinical symptoms, and the condition was aggravated, which represented an ineffective case. The surgical efficacy was calculated as effective cases/total number of cases × 100%.

The complications and treatment satisfaction of the patients were observed and recorded. Complications are infection, arthritis, etc. Satisfaction was evaluated by satisfactory, approximate satisfactory, and dissatisfactory, and treatment satisfaction was calculated by (satisfactory + approximate satisfactory)/total cases × 100%.

### 2.5. Statistical Analysis

Statistical software SPSS20.0 was used for data analysis. Categorical variables were expressed as numbers and percentages and continuous variables as means ± standard deviations, and for comparisons involving three or more groups, one-way analysis of variance (ANOVA) with post hoc Tukey's test for multiple comparisons was employed. The difference was statistically significant (*P* < 0.05).

## 3. Results

### 3.1. Comparison of Ankle Range of Motion

There was no significant difference in ROM among the three groups before treatment (*P* > 0.05), and ROM at 6 months and 12 months after treatment was higher than that before treatment (*P* < 0.05). ROM of group 2 and group 3 was higher than that of group 1 (*P* < 0.05). There was no significant difference between group 2 and group 3 (*P* > 0.05), as shown in Table 2.

### 3.2. Comparison of Ankle Joint Function

There was no significant difference in AOFAS score among the three groups before treatment (*P* > 0.05), and the AOFAS scores at 6 months and 12 months after treatment were higher than that before treatment (*P* < 0.05). The AOFAS scores of group 2 and group 3 were higher than that of group 1 (*P* < 0.05). There was no significant difference between the two groups (*P* > 0.05), as shown in Table 3.

### 3.3. Comparison of Ankle Pain in Patients

There was no significant difference in VAS score among the three groups before treatment (*P* > 0.05), and the VAS scores decreased at 6 months and 12 months after treatment (*P* < 0.05). The VAS scores of group 2 and group 3 were lower than that of group 1 (*P* < 0.05). There was no significant difference between group 2 and group 3 (*P* > 0.05), as shown in Table 4.

### 3.4. Comparison of Surgical Efficacy of Patients

The surgical efficacy of group 2 and group 3 was higher than that of group 1 (*P* < 0.05), and there was no significant difference between the two groups (*P* > 0.05), as shown in Table 5.

### 3.5. Comparison of Postoperative Complications and Treatment Satisfaction of Patients

There was no significant difference in the complication rate among the three groups (*P* > 0.05). The treatment satisfaction of group 2 and group 3 was higher than that of group 1 (*P* < 0.05), and there was no significant difference between the two groups (*P* > 0.05), as shown in Table 6.

## 4. Discussion

At present, the clinical research on the mechanism of talus osteochondral injury is relatively clear with complete classification. However, due to the fracture severity and different treatment methods, there are still differences in prognosis effect and long-term efficacy [5]. It is difficult to repair the defect part of Hepple V talus osteochondral injury. According to Hepple stage, conservative therapy is the preferred treatment for stage III and previous injury treatment, while surgery is required for stage III to stage V [6, 7]. Since there is bone cyst formed in Hepple V talus osteochondral injury, conservative therapy alone brings no effect. Currently, surgery is often used for the treatment of this disease, but the research on the choice of surgical procedure for treatment has always been controversial [8].

The three different surgical procedures used in this study are microfracture surgery, osteochondral autologous transplantation, and periosteal iliac bone transplantation, each of which has its own advantages and disadvantages [9]. Microfracture surgery can stimulate bone marrow mesenchymal stem cells to transform into chondrocytes and repair fibrocartilage, which can effectively improve the clinical symptoms or delay the progression of ankle joint degeneration [10]. However, the effect is not so good in the case of large area injury or bone cyst of Hepple V talus osteochondral injury [11]. The advantages of osteochondral autologous transplantation lie in the use of hyaline cartilage to repair the lesion, and its biomechanical characteristics are very similar to the surrounding normal cartilage. However, pain in the bone donor site occurs occasionally [12, 13]. Periosteal iliac bone transplantation can transform into chondrocytes through periosteal cartilage metaplasia, further promote the healing of cartilage and metatarsal cartilage, and form a whole with subperiosteal bone after differentiation into cartilage, avoiding stratification. The donor site of iliac bone is larger, and the advantage is prominent for large area injury [14].

The data of this study showed that there was no significant difference in ROM, AOFAS score, and VAS score before treatment (*P* > 0.05). After 6 months and 12 months of treatment, ROM and AOFAS score of group 2 and group 3 were higher than those of group 1, and VAS score was lower than that of group 1, indicating statistical significance. The results suggested that osteochondral autologous transplantation and periosteal iliac bone transplantation can effectively remove the lesions and fill them accurately, which can not only ensure the mechanical orientation through structural support but also provide an ideal environment for cartilage repair. Although the effect of group 1 was worse than that of group 2 and group 3, the improvement was significant compared with that before treatment. There was no significant difference in ROM, AOFAS score, and VAS score between the two groups at 6 months and 12 months after treatment (*P* > 0.05). The results indicated that osteochondral autologous transplantation and periosteal iliac bone transplantation have similar effects on improving ankle joint range of motion, promoting ankle function recovery, and alleviating ankle joint pain. The results of this study showed that there was no significant difference in the complication rate among the three groups (*P* > 0.05). The results indicated that the three surgical procedures were safe. The results indicate that the three surgical methods are safe. The surgical efficacy and treatment satisfaction of group 2 and group 3 were higher than that of group 1, indicating statistical significance (*P* < 0.05). However, there was no significant difference in the surgical efficacy and treatment satisfaction of the above two methods (*P* > 0.05). The results suggested that the surgical efficacy of osteochondral autologous transplantation and periosteal iliac bone transplantation are almost the same. In summary, in the treatment of patients with Hepple V talus osteochondral injury, microfracture surgery is appropriate for superficial or small diameter bone cysts; osteochondral autologous transplantation or periosteal iliac bone transplantation should be selected for deep and large-diameter bone cysts according to the actual situation of patients [15].

In conclusion, all the three different surgical procedures for Hepple V talus osteochondral injury have good therapeutic effect. However, osteochondral autologous transplantation and periosteal iliac bone transplantation have better effect in reducing ankle joint pain and promoting ankle joint function recovery, which can effectively improve the treatment satisfaction of patients. Therefore, it is suggested that the selection of surgical procedures should be flexible according to the actual situation of patients. But this study also has its limitation as it only included 60 patients with Hepple V talus osteochondral injury admitted to our hospital from January 2020 to January 2021. We have ignored the long-term effect of different surgical procedures, and we will fullfill this problem in our further study.

## Figures and Tables

**Table 1:** Comparison of basic data of patients.

Group	No. of cases	Gender (*n*, %)		Age range	Average age
		Male	Female		
Group 1	17	11 (64.71%)	6 (35.29%)	30–48	38.20 ± 0.80
Group 2	20	12 (60.00%)	8 (40.00%)	30–49	38.10 ± 0.90
Group 3	23	11 (47.83%)	12 (52.17%)	30–50	38.00 ± 1.00
*P*	/	0.530		0.651	

**Table 2:** Comparison of ankle range of motion.

Group	No. of cases	Before treatment	6 months after treatment	12 months after treatment
Group 1	17	45.45 ± 7.17	54.25 ± 5.00^a^	59.94 ± 5.27^a^
Group 2	20	45.48 ± 7.15	60.25 ± 5.10^ab^	63.60 ± 5.30^ab^
Group 3	23	45.43 ± 7.19	63.90 ± 5.00^ab^	65.95 ± 5.10^ab^

Note: Compared with that before operation, ^a^*P* < 0.05; compared with group 1, ^b^*P* < 0.05.

**Table 3:** Comparison of ankle joint function of patients.

Group	No. of cases	Before treatment	6 months after treatment	12 months after treatment
Group 1	17	71.39 ± 4.51	80.12 ± 3.10^a^	87.88 ± 3.80^a^
Group 2	20	70.41 ± 4.52	88.82 ± 3.00^ab^	91.02 ± 3.30^ab^
Group 3	23	70.43 ± 4.47	88.80 ± 3.04^ab^	88.80 ± 3.04^ab^

Note: Compared with that before operation, ^a^*P* < 0.05; compared with group 1, ^b^*P* < 0.05.

**Table 4:** Comparison of ankle pain in patients.

Group	No. of cases	Before treatment	6 months after treatment	12 months after treatment
Group 1	17	7.89 ± 1.05	4.20 ± 1.00^a^	3.59 ± 0.78^a^
Group 2	20	7.91 ± 1.03	3.05 ± 0.80^ab^	2.50 ± 0.89^ab^
Group 3	23	7.90 ± 1.04	3.02 ± 0.75^ab^	2.45 ± 0.80^ab^

Note: Compared with that before operation, ^a^*P* < 0.05; compared with group 1, ^b^*P* < 0.05.

**Table 5:** Comparison of ankle pain in patients.

Group	No. of cases	Effective	Ineffective	Surgical efficacy
Group 1	17	12 (70.59%)	5 (29.41%)	12 (70.59%)
Group 2	20	19 (95.00%)	1 (5.00%)	19 (95.00%)^a^
Group 3	23	22 (95.65%)	1 (4.35%)	22 (95.65%)^a^

Note: Compared with group 1, ^a^*P* < 0.05.

**Table 6:** Comparison of postoperative complications and treatment satisfaction (*n*, %).

Group	No. of cases	Complication rate	Satisfaction
Group 1	17	0 (0.00%)	12 (70.59%)^a^
Group 2	20	0 (0.00%)	19 (95.00%)^a^
Group 3	23	0 (0.00%)	22 (95.65%)^a^

Note: Compared with group 1, ^a^*P* < 0.05.

## Data Availability

The data used to support this study is available from the corresponding author upon request.
